# The Biomechanics of Shoulder Movement with Implications for Shoulder Injury in Table Tennis: A Minireview

**DOI:** 10.1155/2021/9988857

**Published:** 2021-05-08

**Authors:** Liang Li, Feng Ren, Julien S. Baker

**Affiliations:** ^1^Faculty of Sports Science, East China Jiaotong University, China; ^2^Faculty of Sports Science, Ningbo University, China; ^3^Department of Sport, Physical Education and Health, Hong Kong Baptist University, Kowloon Tong, Hong Kong

## Abstract

A high proportion of shoulder injuries in table tennis players are common, which is both a diagnostic and therapeutic challenge. An understanding of the interaction between biomechanical function of the shoulder and mechanisms of shoulder injuries in table tennis players is necessary to prevent injury and to conduct clinical treatment of the shoulder as soon as possible. The purpose of this minireview was to select the available evidence on the biomechanical characteristics of shoulder movement and potential relationships with various shoulder injuries that are common in table tennis players. Five studies revealed interesting biomechanical characteristics of shoulder movement patterns in table tennis players: large internal rotation torque, an increased torsion-rotation movement, and a greater angular velocity of internal rotation were found. Two studies were noted that were related to specific shoulder injury: glenohumeral internal rotation deficit (GIRD) and impingement syndrome. Unfortunately, it is difficult to draw conclusions on the mechanisms of shoulder injury in table tennis players due to the little evidence available that has investigated shoulder injury mechanisms based on biomechanical characteristics. Future studies should focus on the potential relationship between the biomechanical characteristics of the shoulder and injury prevalence to provide valuable reference data for clinical treatment.

## 1. Introduction

Table tennis as a racket sport is composed of diverse attacking and defensive stroke techniques that demand high muscular strength, movement flexibility, and body coordination. To reach a competitive level, the dynamic exchange of intricate strokes and versatile tactics is necessary to achieve high spins and high velocities of the ball [1]. Players also need to perform aggressive maneuvers with emphasis on power and acceleration conducted repetitively throughout the training session [1]. The long-duration practice and repetitive stress along with the intensive loading sequences create asymmetrical muscle work, leading to overload at particular joints eventually causing injury and deformations. A retrospective study showed that one-fifth of table tennis players suffered from shoulder injuries, and epidemiological data on table tennis players from Slovenia indicated that 20% of injuries were located at the shoulder, followed by 15% in the hip, 13% in the ankle, and 11% in the wrist [2].

The shoulder joint is the principal contributor to energy transfer in table tennis players [3]. From the motor function analysis, the shoulder is the most flexible joint in the human body, which provides anatomical stability allowing for a wide range of motion (ROM) in different directions. However, this kind of biomechanical characteristic causes a fragile equilibrium between stability and mobility, particularly in table tennis players, who require a high level of muscle activity around the shoulder joint to produce as much strength and force as possible to impact the ball. If the scapula fails to conduct its stabilization role, this may lead to a decreased level of performance but also result in shoulder injury [4]. Specifically, scapula impingement syndrome is commonly found in table tennis players, which may be caused by the high loading in the glenohumeral and scapulothoracic joint during table tennis movements [5–8]. The clinician and sports physician should have a comprehensive knowledge of the biomechanical mechanics of the shoulder joint in table tennis players. A review has shown typical characteristics of shoulder joint activity in elite athletes whose greater maximum ROM of shoulder internal rotation and a larger shoulder joint torque in the coronal plane were found when compared to those of low-level players, and these features are strongly related to the performance level of a player [3]. A previous study had already emphasized that excessive loading of a segment is the main factor contributing to a high risk of injury [9].

However, there were no articles reviewed that focused on shoulder injury and its relationship with the biomechanical characteristics of shoulder movement and injury during table tennis performance. Injury mechanics is an important prerequisite for conducting injury prevention as well as clinic treatments. Therefore, it is necessary to reveal and examine the relationship between the mechanical origin of shoulder injuries and shoulder movements in table tennis players. The objective of this review was to summarize the biomechanical characteristics of shoulder movement in table tennis players and to explore its potential relationship with shoulder injury.

## 2. Methods and Material

The approach of relevant literature searching was conducted following the suggestion of the PRISMA (Preferred Reporting Items for Systematic Reviews and Meta-Analyses) statement. Common electronic databases were used for collecting published papers after 2008, which included PubMed, Scopus, Web of Science, and Embase. The manual search was performed on 13 January 2021. The following keywords were used for the search strategy: sport (“table tennis”), injury type (“injury” or “sports injury” or “disease” or “pathology” or “shoulder injury” or “upper extremely injury” or “impingement syndrome” or “glenohumeral internal rotation deficit”), and population (“male” or “female” and “adult”). These words were searched in different combinations on each database. During this process, the collected articles were screened by the first and second authors independently. Preliminary data collection was mainly dependent on the article title, abstract, and language.

### 2.1. Eligibility Criteria and Article Selection

The articles were retrieved using the following inclusion criteria, which were used for identifying articles that were eligible for the study:

- A shoulder injury in table tennis adult players
- The movement skills including the “topspin forehand” and “topspin backhand”
- Biomechanical analysis on table tennis movement
- Articles published in English scientific journals that were peer-reviewed
- The paper being retrievable
- The number of the participant sample size larger than *N* = 6

### 2.2. Quality Assessment

The validated assessment of the retrieved articles was evaluated based on the principle of the McMaster Critical Review Form. This guideline can be used to determine the validity of the assessment study. The criteria are related to 15 dichotomous questions; each question was assigned 1 point to estimate the quality of the selection study, there are two different criteria, including “yes” (1 point) and “no” or “not measured” (0 point) [10], and details of the quality evaluation of the article are shown in Table 1. If there was any disagreement in the process of quality assessment, the authors consulted with each other to reach a consensus for each article reviewed.

## 3. Result

443 articles were found via manual searching on electronic databases, and by selecting articles that complied with inclusion criteria, 7 studies were considered for review. Details of screening the qualified articles are provided in Figure 1.

During the movements involved in the topspin forehand, elite table tennis players exerted a significantly larger torque for shoulder internal rotation than intermediate players to produce a high racket speed during an attacking shot [3]. One article noted that the internal rotation of the shoulder joint plays an important role in the coordination of the forehand stroke, which increased angular velocity of the arm and then influenced the racket velocity. Meanwhile, during the backhand stroke, the larger ROM of the shoulder girdle rotation was directly correlated with the racket velocity [11]. Another research paper emphasized the importance of a shoulder movement strategy in table tennis. It was noted that the relationship between maximal shoulder extension and the maximum velocity of the racket at impact suggested that torsion-rotation movement of the shoulder could be useful in visual training to predict the players' performance level [12]. It has also been confirmed that there are significantly increased angular velocities during shoulder internal rotation when receiving topspin and backspin drives [13]. On the other hand, Iino et al. investigated the shoulder function when transferring the mechanical energy in the racket arm by using inverse dynamics, and they found that shoulder joint force and torque were the largest contributor to energy transfer during both topspin and backspin strokes [14].

Regarding the potential risk of impingement syndrome in table tennis athletes, Meghdadi et al. considered the muscle activity patterns of the shoulder girdle component at the movement of forehand topspin and noted that the ROM of the shoulder girdle muscles which included scapulothoracic and glenohumeral joints were changed in the player who experienced shoulder impingement syndrome [15]. Additionally, Kamonseki et al. explored the occurrence of glenohumeral internal rotation deficit in the dominant shoulder of table tennis players, and results presented a decreased internal rotation in the dominant shoulder compared to the nondominant side [16]. Article details are presented in Table 2.

## 4. Discussion

The shoulder muscle has been considered one of the most vulnerable anatomical muscles in table tennis players. This results from the abrupt and fast movement in a repetitive way during long-term training and match sessions. In particular, a high injury risk of the shoulder is common in elite or professional players, and 20% of injuries of the shoulder were reported in top Slovenian racket sport players. In this review, we collected relevant reference data and explored the mechanisms of shoulder injury based on the biomechanical features of shoulder movements in table tennis players.

Our results indicate that the biomechanical characteristics of shoulder activity are mainly focused on the movement during the forehand topspin loop. This is one of the most aggressive shots for returning backspin balls at a high racket speed, and it is also an important factor for identifying the performance levels of players. This type of skill places a high demand on shoulder joint movements, such as larger internal rotation torque, an increased torsion-rotation movement, and a greater angular velocity of internal rotation which have been reported on collected studies [17]. These kinematic and kinetic characteristics described for the shoulder joint are considered important positive contributors to generating impact speed for the racket but are also related to potential shoulder injury. An increased ROM of the glenohumeral and scapulothoracic joints could generate extra loading on shoulder girdle muscles [18]. This then poses enormous stress on the ligaments, rotator cuff stabilizing muscle, and tendons, gradually leading to impingement syndrome of the dominant shoulder as well as glenohumeral internal rotation deficit (GIRD) [19].

The mechanism of GIRD has been well demonstrated in throwing sports, and it has been indicated previously that the deceleration phase of a throw is the main reason for GIRD injury, but there is still confusion of how the injury occurs in racket sports [19–21]. In this review, we found only one eligible article related to GIRD of the dominant shoulder in table tennis players. The findings demonstrated a significantly smaller angle of internal rotation in the dominant side than in the nondominant shoulder [16]. The authors assumed that the internal rotation deficit in the dominant shoulder was a result of posterior glenohumeral contracture which was caused by repeating microtrauma during the deceleration phase of the forehand [22]. The authors failed to analyze the inner mechanism of GIRD combining muscle strength and biomechanical features of the shoulder. Regarding the injury mechanism of GIRD in the tennis player, the repetition of abduction-extension movements and overhand strokes changes the rotation arc of the shoulder, increasing external rotation accompanied by a tight posterior capsule, which further decreases the ROM of internal rotation and ultimately leads to the development of GIRD [17]. Different from throwing sports, table tennis does not have a throwing motion; the adaptations to the shoulder muscles are different between different table tennis movements. Therefore, the mechanical origin of GIRD in table tennis using specific movements should be explored in the future. This is crucial for clinicians to familiarize themselves with the pathology, diagnosis, and treatment of table tennis shoulder injuries.

Additionally, impingement syndrome is also common in racket players, which is identified as the abnormal impingement and continual compressive force in the glenohumeral joint [23]. Meghdadi et al. observed the dysfunction of shoulder muscles in table tennis players with impingement syndrome, in which the activation and recruitment sequence of shoulder muscles were disordered, and the activity level of the serratus anterior and supraspinatus muscle was significantly reduced [15]. Similarly, additional research confirmed that the activity level of the serratus anterior muscle was decreased in an impingement syndrome group [24]. Specifically, the lower level of activity in the serratus anterior muscle contributes to an abnormal movement of the scapula, which is the main factor for developing impingement syndrome [25]. Meanwhile, the limitation of normal posterior inclination and upward rotation of the scapula may lead to more impingement on the rotator cuff tendons [26]. High levels of muscular control are needed to constantly maintain the stability of the shoulder joint during table tennis performance. One selected studies reported different levels of normalized concentric and eccentric muscular activity using electromyography (EMG) during the movement of forehand topspin [15]. A larger concentric internal rotation of the shoulder is required in forehand servers, which would cause more muscular imbalance between the posterior rotator cuff and internal rotators [27]. Several studies noted that the balance of muscle strength around the shoulder girdle and the correct sequence time of recruiting scapular and rotator cuff muscles are important factors for the stability of glenohumeral joint function and the coordinated motion of the shoulder joint [25, 28]. An inappropriate position of the shoulder components and the dysfunction of the shoulder girdle muscles pose a high risk of subacromial swelling and other related anatomical damage to the shoulder joint [29–32].

## 5. Conclusion

The motion of the shoulder joint during table tennis strokes presents a large internal rotation torque, an increased torsion-rotation movement, and a greater angular velocity of internal rotation, which are the typical biomechanical characteristics of shoulder movement in table tennis. Conducting these repetitive activities for long periods would cause overload stress and microtrauma to musculoskeletal tissues associated with the shoulder joint. At present, unfortunately, there are few studies investigating shoulder injury in table tennis players. The poor localization and diagnosis of shoulder dysfunction in table tennis players often delay timely intervention and rehabilitation. The prerequisite for effective prevention and treatment of injuries is based on a better understanding of the factors that contribute to the injury. Therefore, the potential relationship between biomechanical characteristics and shoulder injuries should be explored in future experimentation, to provide a valuable reference point for clinical treatments and medical interventions.

## Figures and Tables

**Figure 1:** Procedure of the systematic search and selection.

**Table 1:** Methodological quality of included studies by using the McMaster critical appraisal form.

References	Study design	Level	Items															Score
			1	2	3	4	5	6	7	8	9	10	11	12	13	14	15	
[3]	CCT	III-2	√	√	√	√	√	√	x	√	n/a	√	√	√	√	x	√	12/14
[11]	CCT	III-2	√	√	√	√	√	√	√	√	n/a	√	√	√	√	x	√	13/14
[12]	CCT	III-2	√	√	√	√	√	x	√	√	n/a	√	√	√	√	√	√	13/14
[13]	CCT	III-2	√	√	√	√	√	√	√	√	n/a	√	√	√	√	x	√	13/14
[14]	CCT	III-2	√	√	√	√	√	√	√	√	n/a	√	√	√	√	x	√	13/14
[15]	CCT	III-2	√	√	√	√	x	x	√	√	n/a	√	√	√	√	x	√	11/14
[16]	CCT	III-2	√	√	√	√	√	√	√	√	n/a	√	√	√	√	x	√	13/14

Level of evidence (based on NHMRC hierarchy). CCT = control clinical trial; FU/RCT = follow-up study from randomized control trial; √ = yes; x = no/not reported; n/a = not applicable. McMaster items: 1—study purpose clearly stated; 2—background literature reviewed; 3—appropriate research design; 4—sample described in detail; 5—sample size justified; 6—outcome measurer reliability reported; 7—outcome measurer validity reported; 8—intervention described; 9—contamination avoided; 10—cointervention avoided; 11—results reported in terms of statistical significance; 12—appropriate analysis method; 13—clinical significance reported; 14—dropouts reported; 15—appropriate conclusion.

**Table 2:** Summary of the collection of articles.

References	Number of subjects	Main parameter	Comparison	Movement type	Main result related to the shoulder
Iino and Kojima [3]	18	Forces and torques at the shoulder joint	Advanced vs. intermediate player	Forehand stroke	Larger shoulder internal rotation torque in an advanced player
Bańkosz and Winiarski [11]	10	Angular velocities and ROM at the shoulder	Topspin forehands vs. topspin backhands	Topspin forehand and topspin backhand	Larger angular velocity of internal arm rotation and adduction in the shoulder joint at topspin backhands
Malagoli et al. [12]	10	Angular velocities and ROM at the shoulder	Crosscourt vs. long line	Topspin shot	Maximal shoulder extension related to maximum velocity of the racket at impact
Tsai et al. [13]	5	Angular velocities	**—**	Topspin and backspin serves	Elite player increased shoulder external rotation angular velocity in receiving topspin and backspin serves
Iino and Kojima [14]	10	Joint kinetics at the shoulder	**—**	Topspin backhand	Energy transfer by the shoulder joint force in the vertical direction was the largest
Meghdadi et al. [15]	60	EMG	Shoulder impingement syndrome vs. without shoulder impingement syndrome	Forehand topspin loop	Impingement syndrome correlated with disturbed timing and activity level of shoulder girdle muscles
Kamonseki et al. [16]	20	Motion of internal and external rotation and total rotation motion of the glenohumeral joint	Dominant vs. nondominant shoulders	**—**	The dominant side showed decreased internal rotation

## Data Availability

The data that support the findings of this study are available from the corresponding author upon reasonable request.
